The article "A Prognostic Model for the Respiratory Function of Patients with Nonsevere Pulmonary Infection Based on Breathing Exercises and Acupuncture Therapy: Development and Validation" was published in 2022. Journal: Comput Math Methods Med.

# A Prognostic Model for the Respiratory Function of Patients with Nonsevere Pulmonary Infection Based on Breathing Exercises and Acupuncture Therapy: Development and Validation

**DOI:** 10.1155/2022/9057575

**Published:** 2022-09-29

**Authors:** Yulin Shi, Yong Hu, Guomeng Xu, Yaoqi Ke

**Affiliations:** ^1^Department of Rehabilitation Medicine, Xiangyang Central Hospital, Affiliated Hospital of Hubei University of Arts and Science, China; ^2^Department of Respiratory Medicine, Xiangyang Central Hospital, Affiliated Hospital of Hubei University of Arts and Science, China

## Abstract

**Objective:**

In this study, a prognostic model for the respiratory function was constructed based on the treatment methods of patients with nonsevere pulmonary infection, aiming to provide a reference for clinical decision-making.

**Method:**

A total of 500 patients with nonsevere pulmonary infection were included in this study. The patients were randomized into training set (*n* = 350) and validation set (*n* = 150), and the baseline characteristics were collected. All patients received breathing exercises or breathing exercises combined with acupuncture therapy for 3 months, and then the forced expiratory volume in one second (FEV1)/forced vital capacity (FVC) was assessed. Next, an ordinal multinomial logistic regression model was used to analyze prognostic factors affecting respiratory function of patients with nonsevere pulmonary infection. The Test of Parallel Lines was used to determine the accuracy (ACC) of the model and screen the influencing factors. The confusion matrix was drawn, and the ACC and harmonic mean (F1 score) were calculated to evaluate the feasibility of the model results.

**Results:**

Results of the ordinal multinomial logistic regression model showed that age (*P* = 0.000), treatment method (*P* = 0.000), underlying diseases (*P* < 0.001), and sex (*P* = 0.389) were independent factors affecting the respiratory function of patients in the training set. The ACC value of the training set was 88.86%, and that of the validation set was 91.33%, indicating a high accuracy and favorable predictive ability of the model. Besides, the F1 score was 62.38%, indicating a high reliability of the model.

**Conclusion:**

The prognostic model for respiratory function of patients with nonsevere pulmonary infection constructed in this study had favorable predictive performance, which is of great significance in the clinical nursing and treatment of patients with pulmonary infection.

## 1. Introduction

Pulmonary infection generally refers to bacterial, fungal, or viral infection in the lungs or pulmonary parenchyma, resulting in a series of inflammatory reactions [1]. Pneumonia patients show a variety of clinical symptoms, among which the most typical one is dyspnea. Dyspnea patients cannot smoothly breathe with asthma of varying severity, shortness of breath, and even gasp [1]. It was demonstrated that patients with pulmonary infection generally have a favorable prognosis when they receive timely treatment [2]. Breathing exercises are often used to help patients with pulmonary infection recover the respiratory function and improve their quality of life.

The article "A Prognostic Model for the Respiratory Function of Patients with Nonsevere Pulmonary Infection Based on Breathing Exercises and Acupuncture Therapy: Development and Validation" was published in 2022. Journal: Comput Math Methods Med.

Breathing exercises can mend ventilation, improve diaphragmatic function, endurance, and coordination, and maintain or improve thoracic motion, thereby helping to establish effective breathing patterns and relieve respiratory diseases [3]. As a common clinical nursing method, breathing exercises are widely used. For example, the incidence of postoperative pulmonary complications after laparoscopic colorectal surgery can be reduced by perioperative breathing exercise [4]. Charususin et al. [5] demonstrated that breathing exercise can improve the respiratory function of patients with chronic obstructive pulmonary disease (COPD). However, a randomized trial shows no significant improvement in the respiratory function of patients with COPD after exercise-training plus breathing-retraining [6]. Furthermore, acupuncture, as a unique Chinese therapy, is a kind of medical skill of “internal diseases treated by external application” which is also widely used in clinical treatment of lung diseases to decrease adverse symptoms such as dyspnea. A study indicated that warm acupuncture plays an effective role in the improvement of symptoms of patients with acute exacerbation COPD with phlegm-turbid obstruction of the lung [7]. A systematic review illustrated that acupuncture may remarkably improve dyspnea and quality of life of patients [8]. Hence, we constructed a prognostic model for the respiratory function based on breathing exercises and acupuncture therapy, thereby investigating the prognostic factors affecting the respiratory function of patients with nonsevere pulmonary infection.

The study of pneumonia prognosis is of notable value. Ahn et al. [9] constructed a prognostic model for patients with pneumonia, confirming that Eastern Cooperative Oncology Group (ECOG) scores, oxygen saturation (SpO_2_), and lactic acid are independent prognostic factors of mortality. Another research constructed a COX proportional-hazards model to analyze the mechanical ventilation prognosis of patients with hypoxemic acute respiratory failure treated with high-flow nasal cannula (HFNC) [10]. In this study, we constructed an ordinal multinominal logistic regression model with the baseline characteristics of patients as input variables, used parallel line hypothesis to determine the accuracy of the model, screened the influencing factors, drew confusion matrices, and calculated the prediction accuracy of the model.

The article "A Prognostic Model for the Respiratory Function of Patients with Nonsevere Pulmonary Infection Based on Breathing Exercises and Acupuncture Therapy: Development and Validation" was published in 2022. Journal: Comput Math Methods Med.

## 2. Materials and Methods

### 2.1. Subject

Clinical data of 500 patients with nonsevere pulmonary infection treated in our hospital were collected in this study. The inclusion criteria for patients were CURB (confusion, uremia, elevated respiratory rate, and hypotension) score ≤ 2, consciousness disorders, urinary nitrogen ≥ 7 mmol/L, respiratory rate ≥ 30 times/min, systolic pressure ≤ 90 mmHg or diastolic blood pressure ≥60 mmHg, and age ≥ 65. Patients with serious underlying diseases were excluded.

All patients were divided into training set (*n* = 350) and validation set (*n* = 150) by random sampling method. The training set was utilized to construct the model and the validation set was employed to verify the accuracy of the prognostic model. Breathing exercise mainly referred to two maximal continuous ventilation maneuvers per day for 15 min with a 15-min interval between the two maneuvers. Breathing exercise combined with acupuncture therapy was performed twice a week for 10 min each on the basis of breathing training. The cycles for both treatments were 3 months. Manifested in Table 1 are clinical characteristics of the two groups. The study received ethical approval from the Ethics Committee of Xiangyang Central Hospital, Affiliated Hospital of Hubei University of Arts and Science. Since this was a retrospective study, the informed consent of patients was waived.

### 2.2. Prediction of Results

The analysis of qi and blood was performed on the patients before treatment, and partial arterial oxygen pressure (PaO_2_), partial pressure of carbon dioxide (PaCO_2_), and pH of the patients were measured and included as variables affecting respiratory function. Forced expiratory volume in one second (FEV1), forced vital capacity (FVC), and FEV1/FVC ratio were measured after three months of treatment. FEV1/FVC was used as the evaluation index and was divided into three categories according to the diagnosis and classification criteria of GOLD2013 edition. FEV1/FVC < 0.7 was classified as category 1, and 14 patients in this category still had chronic obstructive pulmonary diseases. 0.7 ≤ FEV1/FVC < 0.8 was classified as category 2, and there were 266 patients in total who recovered better. 0.8 ≤ FEV1/FVC < 8 was classified as category 3, and there were 220 patients in total. The respiratory function of these patients had even reached a good level.

### 2.3. Statistical and Analysis

SPSS 26.0 software was used to test the statistical differences of baseline characteristics between two groups. Median (P25, P75) was used for statistical description of measurement data that did not conform to normal distribution. *U*-test was applied for intergroup comparison, while chi-square test was used for intergroup comparison of categorical data. *P* value less than 0.05 was considered statistically significant. Patients were randomly divided into validation set and test set by ‘sample' package of R software, with the ratio of 7 : 3.

The article "A Prognostic Model for the Respiratory Function of Patients with Nonsevere Pulmonary Infection Based on Breathing Exercises and Acupuncture Therapy: Development and Validation" was published in 2022. Journal: Comput Math Methods Med.

The principle of ordinal multinomial logistic regression is that the multiple categories of dependent variable are successively divided into multiple binary logistic regressions. In this study, the FEV1/FVC index was selected, and the dependent variable was three categories with an order relation between the categories. In the analysis, it was divided into two binary logistic regressions, namely (1 vs. 2 + 3) and (1 + 2 vs. 3), both of which contrasted lower level with higher level, and its mathematical Formula (1) was

(1) $$\begin{array}{c} \ln\left[\overset{j}{\underset{i=1}{\sum }}p_{i}\backslash \left(1-\overset{j}{\underset{i=1}{\sum }}p_{i}\right)\right]=a_{j}+\overset{m}{\underset{i=1}{\sum }}b_{i}x_{i},j=1,2, \end{array}$$

where *X* = (*x*_1_, *x*_2_, ⋯, *x*_*m*_) is the independent variable vector, *p*_*j*_ is the probability estimation of the dependent variable taking *j* level, *a*_*j*_ is the estimate of the intercept parameter, and *b*_*i*_ is the estimate of the partial regression coefficient *β*_*i*_.

In the ordinal multinomial logistic regression model, the hypothesis of equal coefficients of independent variables should be tested by parallel lines. The Test of Parallel Lines is also the process of factor screening. First, the factor selected should make the test *P* (Sig.) value greater than 0.05. In this case, the null hypothesis was not rejected, so the hypothesis could be considered as valid and ordinal multinomial logistic regression can be used. Next, the chi-square (likelihood ratio) test was used to make an overall evaluation of the model, *χ*^2^ = 487.665, *P* = 0.000 indicating that the model was statistically significant. At the same time, by referring to the Pearson's chi-squared test *P* = 1.000 > 0.05 and deviation test *P* = 1.000 > 0.05 for the goodness of fit, model was suggested to be statistically significant.

To screen the remarkable influencing factors of evaluation index, the ordinal multinomial logistic regression model was gradually established in the direction of the increase of *P* (Sig.) value assumed by parallel lines. The *P* value of the full variable model before screening was 0.000, and the *P* value of the optimal model after screening was 0.816, with *P* > 0.05 in the results, so the null hypothesis was accepted. The results of optimal multinomial ordered logistic regression are shown in Table 2. Age (*P* = 0.000), treatment method (*P* = 0.000), underlying diseases (*P* < 0.001), and sex (*P* = 0.389) were independent factors affecting the respiratory function of patients in the training set.

The article "A Prognostic Model for the Respiratory Function of Patients with Nonsevere Pulmonary Infection Based on Breathing Exercises and Acupuncture Therapy: Development and Validation" was published in 2022. Journal: Comput Math Methods Med.

An ordinal multinomial logistic regression was constructed. The Test of Parallel Lines was used to determine the accuracy [11] of the model and screen the influencing factors. The confusion matrix was drawn, and the accuracy (ACC) of predicted result by the model (ACC, Formula (2)) as well as the harmonic mean (F1 score, Formula (3)) was calculated.

(2) $$\begin{array}{c} \text{ACC}=\frac{\text{TP}+\text{TN}}{\text{TP}+\text{FN}+\text{FP}+\text{TN}}, \end{array}$$

(3) $$\begin{array}{c} F_{1}=\frac{2\times P\times R}{P+R}, \end{array}$$

where TP is the true positive, TN is the true negative, FP is the false positive, FN is the false negative, *P* is the Precision, and *R* is the recall.

## 3. Results

### 3.1. Clinical Characteristics of Patients

In the training set, the age distribution of patients was 54 (45, 65) years old, including 174 males (49.7%) and 176 females (50.3%), and 171 patients (48.9%) with only breathing exercises and 179 patients (51.1%) with combined breathing exercise and acupuncture therapy. In the validation set, the age distribution of patients was 56 (45, 67) years old, including 74 males (49.3%) and 76 females (50.7%), and 78 patients (50.7%) with only breathing exercises and 72 patients (48%) with combined breathing exercise and acupuncture therapy. Other baseline characteristics are shown in Table 1.

### 3.2. Construction of an Ordinal Multinomial Logistic Regression Model

The Estimates of Stage = 1 and 2 corresponding to threshold were the constant terms of the two binary logistic regressions split in this analysis. The parameter Estimate (-0.047) corresponding to the age was the Estimate of the independent variable.

-4.754 of the treatment = 0 coefficient (Estimate) indicated that patients treated with breathing exercise alone were at least 12.922 times more likely to recover at least one grade higher respiratory function than those treated with breathing exercise combined with acupuncture under certain variables [exp (-4.754)], indicating that respiratory training combined with acupuncture therapy had a better recovery effect. The other coefficients were interpreted the same way.

The sex variable coefficient presented no statistical significance (*P* = 0.389). However, this study considered age affecting respiratory function. Even in this study, its coefficient was not significant and it should be retained in the model (because no statistical significance might be caused by small sample size, and it did not mean the variable had no effect). Therefore, it was retained in this study.

The article "A Prognostic Model for the Respiratory Function of Patients with Nonsevere Pulmonary Infection Based on Breathing Exercises and Acupuncture Therapy: Development and Validation" was published in 2022. Journal: Comput Math Methods Med.

### 3.3. Assessment and Validation of the Model

Confusion matrix diagram (Figure 1) and confusion matrix table for predicted results (Table 3) were drawn based on the constructed optimal multinomial ordered logistic regression model, and then the ACC value of the model was calculated. The ACC value of the training set was 88.86%, and that of the validation set was 91.33%, indicating that the prognostic model of respiratory function in patients with nonsevere pulmonary infection constructed in this study had high ACC. Subsequently, by calculating the recall ratio (63.71%) and precision ratio (61.11%), the F1 score was obtained to be 62.38%, further indicating that the performance of the model was reliable.

## 4. Discussion

In this study, a prognostic model of respiratory function in patients with nonsevere pulmonary infection was constructed based on the treatment methods, which indicted the effects of the age, treatment methods, underlying diseases, and sex on the recovery of respiratory function. The results showed that ACC value of the training set was 88.86%, and that of the validation set was 91.33%, indicating the favorable predictive ability and high credibility of the model, which provided certain references for the treatment of patients with nonsevere pulmonary infection.

A study on the risk of COVID-19 progression showed that old age and complications are the independent risk factors of the progression of pulmonary infection [12]. In recent years, studies on COVID-19 patients have shown that advanced age and comorbidities are susceptible to COVID-19 and increase the proportion of severe cases, which in turn increases the risk of death [13–16]. Singh et al. [17] pointed out that diabetes may worsen the conditions of pulmonary infection. The common underlying diseases of elderly patients mainly include hypertension, coronary heart disease, COPD, diabetes, and cardiovascular and cerebrovascular diseases [14], which may be related to the low immune function in elderly patients. In this study, the results of optimal multinomial ordered logistic regression indicated that the prognosis of respiratory function in elderly patients with pulmonary infection and in patients with underlying diseases is poor. In addition, studies have reported that men are more likely to suffer from COVID-19 [13, 18] and severe acute respiratory distress syndrome [18–20], which may be related to the innate and adaptive immune effects of female sex hormones, although our results showed no statistically significant difference in the effect of sex on respiratory function in patients with nonsevere pulmonary infection, which may be caused by small sample size. Therefore, the clinical management of nonsevere pulmonary infection should comprehensively consider all influencing factors and pay special attention to elderly male patients with underlying diseases.

The article "A Prognostic Model for the Respiratory Function of Patients with Nonsevere Pulmonary Infection Based on Breathing Exercises and Acupuncture Therapy: Development and Validation" was published in 2022. Journal: Comput Math Methods Med.

Breathing exercise was found to help improve COVID-19 symptoms in a randomized controlled trial [21]. Pu et al. [22] demonstrated through meta-analysis that breathing exercise before curative pneumonectomy in lung cancer patients can help reduce hospital length of stay, postoperative pulmonary complications, and pneumonia. In addition, breathing exercise has been confirmed to improve respiratory function and quality of life in patients with COPD and asthma [11, 23, 24]. Acupuncture can also be used as an adjunctive treatment for COPD, asthma, lung cancer, and COVID-19, demonstrating its significant efficacy and safety for respiratory diseases [25–29]. Acupuncture may assist in alleviating symptoms of respiratory diseases by reducing bronchial immune-mediated inflammation and promoting the release of vascular and immune regulatory factors [30]. In this study, a multivariate logistic regression model was constructed to predict respiratory function using FEV1/FVC of patients after treatment as the dependent variable. All patients included in the study underwent breathing exercise or breathing exercise combined with acupuncture for 3 months. The results showed that the respiratory function prognosis of patients with lung infection treated with combined therapy was better than that of patients who underwent breathing exercise alone. However, there were some defects because of the small sample size and the fact that only FEV1/FVC was used as evaluation index of respiratory function.

In conclusion, a prognostic model for respiratory function in patients with nonsevere pulmonary infection was constructed based on the treatment methods, thus obtaining the prognostic impact factors. However, the safety of both treatments was not analyzed in this study. Therefore, more samples should be included in the future, and evaluation indicators should be added based on the optimization of prediction model. Then the impact of breathing exercises and acupuncture therapy on the respiratory function of patients with nonsevere pulmonary infection can be further explored.

## Figures and Tables

**Figure 1:** Confusion matrix diagram of predicted-actual values.

**Table 1:** Comparison of baseline characteristics of patients.

Characteristics	Training set (*n* = 350)	Validation set (*n* = 150)	*P* value
Age (years old)	54 (45, 65)	56 (45, 67)	0.684
Sex			0.938
Male (%)	174 (49.7)	74 (49.3)	
Female (%)	176 (50.3)	76 (50.7)	
Smoking history			0.342
Never (%)	113 (32.3)	42 (28.0)	
Smoking (%)	237 (67.7)	108 (72.0)	
PaO_2_^a^	85 (81, 93)	88.5 (82, 95)	0.784
PaCO_2_^b^	40 (38, 43)	40 (38, 43)	0.600
PH	7.39 (7.37, 7.42)	7.40 (7.37, 7.43)	0.476
Including a least one underlying disease (%)	90 (25.7)	43 (28.7)	0.254
Hypertension (%)	36 (10.3)	23 (15.3)	
Diabetes (%)	34 (9.7)	25 (16.7)	
Hyperlipoidemia (%)	22 (6.3)	19 (12.7)	
COPD (%)	16 (4.6)	14 (9.3)	
Treatment methods			0.520
Breathing exercises only (%)	171 (48.9)	78 (52.0)	
Breathing exercises combined with acupuncture therapy (%)	179 (51.1)	72 (48.0)	

Note: a: partial pressure of oxygen; b: partial pressure of carbon dioxide.

The article "A Prognostic Model for the Respiratory Function of Patients with Nonsevere Pulmonary Infection Based on Breathing Exercises and Acupuncture Therapy: Development and Validation" was published in 2022. Journal: Comput Math Methods Med.

**Table 2:** Parameter estimates of each variable in the ordinal multinomial logistic regression model.

		Estimate	Std. Error	Sig.
Threshold	Stage = 1	-9.501	1.043	0.000
	Stage = 2	15.539	0.817	0.000
Location	Age	-0.047	0.014	0.000
	[treatment = 0]	-4.754	0.445	0.000
	[treatment = 1]	0^a^	.	.
	[underlying disease = 0]	19.980	0.000	< 0.001
	[underlying disease = 1]	0^a^	.	.
	[sex = 0]	0.262	0.304	0.389
	[sex = 1]	0^a^	.	.

treatment = 0: breathing exercise alone; treatment = 1: breathing exercise combined with acupuncture therapy; a: this parameter is redundant and set to 0.

**Table 3:** Confusion matrix of the results predicted by optimal multinomial ordered logistic regression model in the validation set.

Confusion matrix		Predicted category			
		0	1	2	Total number
Actual category	0	0	6	0	6
	1	0	65	0	65
	2	0	7	72	79
	Total number	0	78	72	150

## Data Availability

The datasets generated and analyzed during the current study are not publicly available, but are available from the corresponding author on reasonable request.
